# The Use of Cytotoxic Drugs as First Line Chemotherapy for EGFR (+) Nonsquamous NSCLC: A Network Meta-Analysis

This article has been retracted.

**DOI:** 10.1155/2023/5272125

**Published:** 2023-04-10

**Authors:** Duo Li, Meng Li, Hong Li, Puyu Shi, Mingwei Chen, Tian Yang

**Affiliations:** Department of Respiratory and Critical Care Medicine, The First Affiliated Hospital of Xi'an Jiaotong University, No. 277, West Yanta Road, Xi'an, Shaanxi 710061, China

## Abstract

**Objective:**

To assess the use of cytotoxic drugs as first-line chemotherapy for nonsquamous non-small-cell lung cancer (NSCLC) with EGFR mutation.

**Method:**

This study uses the network meta-analysis (NMA) method, with the inclusion of prospective randomized control studies related to the treatment of EGFR-positive nonsquamous NSCLC, to compare the efficacy of various EGFR-TKIs. As of September 4, 2022, 16 studies on a total of 4180 patients were included. The retrieved literature was comprehensively evaluated as per the established inclusion and exclusion criteria, and valid data were extracted and included for analysis.

**Results:**

The 6 treatment regimens included cetuximab, CTX (cyclophosphamide), icotinib, gefitinib, afatinib, and erlotinib. All of the 16 studies reported their findings about overall survival (OS), and 15 of them also reported findings about progression-free survival (PFS). The NMA results showed that there was no significant difference in OS among the 6 treatment regimens. It was observed that erlotinib had the highest likelihood of obtaining the best OS, followed by afatinib, gefitinib, icotinib, CTX, and cetuximab, in descending order. This indicates that the highest possibility of achieving the best OS was with erlotinib, while the lowest was with cetuximab. The NMA results also showed that the PFS achieved with treatment using afatinib, erlotinib, and gefitinib were all higher than that with treatment using CTX, with statistically significant differences. The results showed that there was no significant difference in PFS among erlotinib, gefitinib, afatinib, cetuximab, and icotinib. CTX, cetuximab, icotinib, gefitinib, afatinib, and erlotinib were ranked in descending order based on the PFS indicator SUCRA values, which implied that erlotinib had the highest possibility in achieving the best PFS, while CTX had the lowest. *Discussion*. EGFR-TKIs must be carefully selected for the treatment of different histologic subtypes of NSCLC. For EGFR mutation (+) nonsquamous NSCLC, erlotinib is most likely to achieve the best OS and PFS, which makes it the first choice in the formulation of a treatment plan.

## 1. Introduction

Non-small-cell lung cancer (NSCLC) is the most common type of lung cancer, accounting for about 80-85% of all lung cancers [1]. Epidermal growth factor receptor (EGFR) is the most prevalently mutated gene in NSCLC, present in about 17% of all NSCLCs, with exonic deletions in chromosomes 19 and 21 being particularly common. EGFR can bind with epidermal growth factors, which are normal protein found in healthy cells taking part in mitosis. However, activating mutation in EGFR can result in constitutive activation of downstream signaling pathways, accelerating abnormal cell growth and proliferation, thus giving rise to carcinogenesis [2]. Several studies have shown that EGFR-TKIs are more effective than standard chemotherapy with regard to PFS and ORR and are increasingly being approved as the first-line treatment for lung cancer [3]. It has been reported that 60% of nonsquamous NSCLC harbor EGFR mutations, the majority of which are found in nonsmokers or former smokers. Most patients with adenocarcinomas or simple squamous cell carcinomas do not have sensitizing EGFR mutations [4, 5].

The treatment of patients with NSCLC not only depends on the histological and genetic subtype of the tumor but also on the stage of disease, comorbidities, and the general condition of the patient. Conventional treatment of NSCLC includes surgery, chemotherapy, radiation therapy, and immunotherapy, yet with undesirable outcomes. In recent years, targeted therapy has received increasing attention. Cytotoxic agents are employed in the traditional pharmacological treatment of NSCLC. With the deepening understanding of EGFR mutations, significant advances have been made in the development of drugs targeting EGFR mutations in lung cancer [6, 7]. Over the past decade, revolutionary changes have taken place in the treatment of patients with EGFR mutation-positive NSCLC owing to the development of EGFR-TKIs, which are considered the first choice for the first-line treatment of this patient population. EGFR-TKIs are a group of drugs that target EGFR mutations, including gefitinib, erlotinib, icotinib, and afatinib [8]. EGFR mutation testing is recommended on patients with nonsquamous NSCLC. Some studies have shown that in comparison to chemotherapy drugs, EGFR-TKIs can significantly prolong the PFS of patients with late-stage NSCLC, despite the lack of a significant difference in OS. EGFR-TKIs should be the first-line treatment for patients with late-stage EGFR-positive NSCLC [9, 10].

NMA conducts weighted and combined analysis based on meta-analysis techniques by combining direct and indirect comparisons of three or more interventions in a single body of evidence. It provides the maximum odds ratio of the model by constructing a hierarchical model that deals with sampling variability, heterogeneity of intervention effects, and inconsistency across studies. NMA can simultaneously compare the treatment effects among multiple interventions in the body of evidence and rank them by treatment effect, thus providing a significant reference for decision makers in the formulation of clinical guidelines. The effectiveness of EGFR-TKIs in nonsquamous NSCLC has already been widely recognized, but there is a lack of studies about the efficacy of various agents in this class of drugs. This study uses the NMA method to compare the efficacy of various EGFR-TKIs, and the results are reported below.

## 2. Materials and Method

### 2.1. Literature Retrieval Strategy

A computer was used for document retrieval from the database, including Cochrane Central Register of Controlled Trials, MEDLINE, Embase, and ISI Web of Science. The search terms included “non-small cell lung cancer”, “NSCLC”, “EGFR-TKIs”, “EGFR mutations”, and “Adenocarcinoma”. Abstracts were excluded, since they do not provide sufficient details for adequate evaluation. The search was limited to the period from the inception of the database to September 4, 2022.

### 2.2. Inclusion and Exclusion Criteria

#### 2.2.1. Inclusion Criteria

1. Patients with biopsy documented adenocarcinoma or large cell carcinoma, TNM stage IIIb or IV
2. EGFR mutation (+) on gene testing
3. At least one group treated with CTX and another with EGFR-TKIs in the intervention measures
4. Randomized control studies
5. Text that includes data on PFS or OS

#### 2.2.2. Exclusion Criteria

1. Dissertations and articles in inappropriate formats, such as review, conference paper, editorial, letter, comment, and note
2. Studies with less than 20 subjects and with a follow-up duration less than 6 months
3. Duplications of previous publications that were superseded by updates
4. Literature published repeatedly
5. The interventions in the treatment and control groups did not meet the aforementioned criteria
6. The study data were poorly described and contained inaccurate information
7. Review, case, case report, and clinical experience-based literature
8. Only experimental animal studies performed on this disease

### 2.3. Data Extraction

Two independent researchers read the articles and extracted the data. When disagreements arose, a third researcher was brought in to make a judgement. Indicators for data extraction included

1. General information: author, year of publication, pathological stage, number of patients, intervention method, follow-up period, etc.
2. Observational indicators: OS, PFS, etc.
3. An email was sent to the author for certain information which could not be obtained from the article. If the author could not be contacted, then it was labeled as “Not Available (N/A)”

### 2.4. Evaluation of Literature Quality

Two researchers assessed the quality of the independent literature, following the guidelines of Cochrane Handbook for Systematic Reviews of Interventions. The quality of the literature was assessed from the following aspects: selective bias, methodological bias, reporting bias, and other potential bias. The literature quality was evaluated according to the criteria with reference to the standard evaluation methods of RCTs, namely, the evidence-based evaluation standard of the Cochrane Medicine Center and the Jadad scale that are used to rate the literature quality of clinical research projects.

### 2.5. Statistical Method

The data was analyzed using R software GeMTC package. The primary indicators of this study are OS and PFS, and the secondary indicators are ORR, AEs, etc. The *I*^2^ test was used to analyze statistical heterogeneity. An *I*^2^ value of 0~24.9% indicates low heterogeneity, and greater values imply increasing heterogeneity (25~49.9%: moderate heterogeneity; 50~74%: substantial heterogeneity; and 75~100%: considerable heterogeneity). The fixed effect model was used for low and moderate heterogeneity, while the random effect model for substantial and considerable heterogeneity. R software was used to draw a bar chart of the surface under the cumulative ranking (SUCRA) and calculate the area under the curve, with the smaller area under the curve indicating the better efficacy.

## 3. Results

### 3.1. General Information of the Included Articles

As shown in Figure 1, the initial search generated 3370 articles, 314 of which were RCT-related articles. After the exclusion of repetitive and unrelated articles, 55 articles were left. Another 39 articles were further excluded owing to its insufficient data and low quality. Thus, a total of 16 articles were left and included in this study. The total number of patients was 4180 (Table 1).

### 3.2. Network Diagrams of the Included Articles

A total of 16 articles reported their findings on OS, including 5 involving erlotinib and CTX, 6 involving gefitinib and CTX, 2 involving afatinib and CTX, 2 involving cetuximab and CTX, and 1 involving icotinib and CTX (Figure 2).

### 3.3. Comparison of Overall Survival (OS)

In the NMA of OS, *I*^2^ = 9%, a fixed effect model was adopted. Compared with CTX, afatinib had an aggregate HR of 0.91 (95% CI: 0.65, 1.30), and the figures for cetuximab, erlotinib, gefitinib, and icotinib were 1.50 (95% CI: 0.81, 2.80), 0.89 (95% CI: 0.67, 1.20), 0.92 (95% CI: 0.74, 1.10), and 0.97 (95% CI: 0.60, 1.60), respectively, all of which indicated no significant difference. In the pairwise comparison with icotinib, erlotinib, gefitinib, afatinib, and cetuximab, no statistical significant difference in OS was observed. The NMA results showed that there was no significant difference in OS among the 6 different agents (Figure 3). As shown in Figure 4, the OS indicator SUCRA values ranked cetuximab, CTX, icotinib, gefitinib, afatinib, and erlotinib in descending order. This shows that erlotinib is most likely to obtain the best OS, while cetuximab is least likely to do so.

### 3.4. Comparison of Progression-Free Survival (PFS)

In the NMA of PFS, *I*^2^ = 18%, a fixed effect model was adopted. Compared to CTX, afatinib, cetuximab, erlotinib, gefitinib, and icotinib revealed an aggregate HR of 0.41 (95% CI: 0.22, 0.75), 1.20 (95% CI: 0.29, 4.80), 0.30 (95% CI: 0.20, 0.46), 0.44 (95% CI: 0.31, 0.62), and 0.61 (95% CI: 0.26, 1.50), respectively. Afatinib, erlotinib and gefitinib significantly improved PFS compared with CTX, and the difference had statistical significance. In the pairwise comparison with erlotinib, gefitinib, afatinib, cetuximab, and icotinib, the results show that there was no significant difference in PFS among the drugs (Figure 5). As shown in Figure 6, the PFS indicator SUCRA values ranked CTX, cetuximab, icotinib, gefitinib, afatinib, and erlotinib in descending order. This implies that erlotinib has the highest probability of obtaining the best PFS, while CTX has the lowest.

## 4. Discussion

In this study, there was no significant difference in the OS between CTX and EGFR-TKIs. Among the EGFR-TKIs, afatinib, erlotinib, and gefitinib had a higher PFS than CTX. Lung cancer is the second most common cause of death worldwide, accounting for 18.4% of all cancer-related deaths. NSCLC is the most common type of lung cancer, with adenocarcinoma accounting for 40% of the cases, followed by squamous cell carcinoma at 25-30% and large cell carcinoma at 5-10% [27]. With the advancement of genetic testing technology, it is now possible to test the circulating tumor DNA by using plasma isolated from peripheral blood. This allows the identification of gene mutations and the formulation of personalized targeted-therapy treatment regimens [28]. Studies have found that 32.9% of NSCLC patients have kinase domain mutations in EGFR, which is shown to be associated with cell growth, proliferation, and migration. It has been suggested that the EGFR gene should be the main target of drugs for lung cancer [29].

Gefitinib, erlotinib, and icotinib are first-generation EGFR-TKIs that can reversibly inhibit EGFR [30]. In the IPASS III study, 1217 patients were divided into two groups; one group was treated with gefitinib, and the other with carboplatin and paclitaxel. The results showed that the PFS of the gefitinib group was higher than that of the chemotherapy group, proving that gefitinib was more effective than chemotherapy, despite the absence of a significant difference in OS [17]. In addition, the OPTIMAL and EURTAC studies [12, 14] that compared the therapeutic effects of erlotinib, carboplatin, and gemcitabine also obtained similar results. The CONVINCE study, which compared the therapeutic effects of icotinib and first-line chemotherapy, found that icotinib can significantly prolong the PFS.

Afatinib is a second-generation EGFR-TKI that can irreversibly inhibit EGFR. The LUX-Lung 3 and LUX-Lung 6 studies [22, 23] compared the therapeutic effects of afatinib and first-line chemotherapy. The results showed that afatinib can significantly prolong the PFS, but there was no significant difference in OS between the two groups. Drug resistance may be one of the causes for the different effects of EGRR-TKIs and CTX on OS and PFS. It is a major problem in cancer treatment and is related to the acquisition of multiple mutations in the neoplastic cells [31, 32]. Treatment using EGFR-TKIs can inhibit growth, proliferation, and migration of neoplastic cells in the early stages. However, with the passage of time, the neoplastic cells acquire new mutations that confer resistance to the effects of EGFR-TKIs. These new mutations either alter the drug target themselves or circumvent tumor dependence on the drug target. This could partly explain why EGFR-TKIs do not have a significant effect on OS [33].

At present, there have been no studies that directly compared the efficacy of various EGFR-TKIs. The drugs that obtained the best OS and PFS in this study were erlotinib, afatinib, gefitinib, and icotinib. This indicates that erlotinib is the best choice of treatment for EGFR (+) nonsquamous NSCLC. For squamous cell lung carcinoma, the LUX-Lung 8 study had different findings. The study included 795 patients with end-stage squamous cell lung carcinoma, who were treated with either erlotinib or afatinib. The results showed that afatinib significantly prolonged OS and PFS compared with erlotinib [34]. Afatinib is a second-generation EGFR-TKI and is more effective in treating squamous cell lung carcinoma than first-generation EGFR-TKIs. Therefore, for different histological types of lung cancer, EGFR-TKIs must be carefully selected [35].

Despite no obvious observed heterogeneity in this study, the following aspects should be considered in the interpretation of the results. Firstly, only 10 of the included studies recruited patients with EGFR mutations, and the rest of the studies were performed on patients with EGFR mutation subgroups, which may have a certain impact on the results. Secondly, there were differences in the use of cytotoxic drugs as first-line chemotherapy in this study, and whether they were combined with chemotherapy in EGFR-TKIs. Thirdly, different studies included patients at different ages, and some of them merely recruited patients over the age of 70. These aspects could exert a certain impact on the outcomes of this study.

This study has limitations in the following aspects: (1) the number of included RCTs was limited, which may lead to biased results; (2) the subjects included in the study were from different countries, which may lead to ethnically biased results; (3) bias analysis was not published owing to the limited literature on the reported indicators analyzed in this study; (4) there was only one study on icotinib, which may result in a weight bias; (5) the quality of the included RCTs was limited, and there was an urgent need for higher-quality RCTs; (6) the data information obtained from the studies was limited, and only overall survival could be obtained, while other survival-related information such as disease-free progression was unclear; and (7) there was certain heterogeneity among the studies.

## 5. Conclusion

For different histological subtypes of NSCLC, EGFR-TKIs should be reasonably selected. In the treatment of nonsquamous NSCLC, erlotinib is the most likely to obtain the best OS and PFS, which makes it the first choice in the formulation of treatment regimens. In clinical practice, the selection of an appropriate targeted drug should not only be based on the mutation type but also on the local medical reimbursement policy and the financial situation of the patient. Despite the promising prospects of sequential treatment with EGFR-TKIs, it is only indicated for NSCLC patients with T790M mutation resistance. If effective molecular diagnostic techniques can be made available soon, the sequential treatment with EGFR-TKIs may become a viable treatment strategy, especially in countries where erlotinib for first-line treatment is limited by cost or other factors. Whether this strategy is more effective than erlotinib as first-line therapy remains an open question and needs to be evaluated in prospective studies.

## Figures and Tables

**Figure 1:** Analysis of the quality of articles included in this study.

**Figure 2:** Network diagram of included articles ((a) is the OS network diagram, (b) is the PFS network diagram). A total of 16 papers presented their findings on OS, including 5 involving erlotinib and CTX, 6 involving gefitinib and CTX, 2 involving afatinib and CTX, 2 involving cetuximab and CTX, and 1 involving icotinib and CTX.

**Figure 3:** NMA forest plot of OS. The differences among erlotinib, gefitinib, afatinib, cetuximab, and icotinib are not statistically significant. The NMA demonstrates that there is no statistically significant change in OS when the six different drugs are employed.

**Figure 4:** Histogram and area of SUCRA in OS. The OS indicator SUCRA values ranked cetuximab, CTX, icotinib, gefitinib, afatinib, and erlotinib in descending order. This demonstrates that erlotinib has the highest chance of achieving the best OS, whereas cetuximab has the lowest.

**Figure 5:** NMA forest plot of PFS.

**Figure 6:** Histogram and area of SUCRA in PFS. The PFS indicator SUCRA values ranked CTX, cetuximab, icotinib, gefitinib, afatinib, and erlotinib in descending order. This demonstrates that erlotinib has the highest chance of achieving the best PFS, whereas CTX has the lowest.

**Table 1:** Articles included in the study.

Author	Year published	Phase	Stage	Total	t1	t2	Mutation
Wu et al. [11]	2015	III	IIIB/IV	217	Erlotinib	CTX	Exon 19 deletion or exon 21 L858R mutation
Rosell et al. [12]	2012	III	III/IV	174	Erlotinib	CTX	Exon 19 deletion or exon 21 L858R mutation
Gridelli et al. [13]	2012	III	IIIB/IV	39	Erlotinib	CTX	Exon 19 deletion mutation
Chen et al. [14]	2012	NA	IIIB/IV	116	Erlotinib	CTX	Exon 19 deletion or exon 21 L858R mutation
Wu et al. [15]	2013	III	IIIB/IV	97	Erlotinib	CTX	Exon 19 deletion, or G719X, L858R, or L861Q mutation
Han et al. [16]	2012	III	IIIB/IV	42	Gefitinib	CTX	Exon 19 deletion or exon 21 L858R mutation
Mok et al. [17]	2009	III	IIIB/IV	261	Gefitinib	CTX	Exon 19 deletion or exon 21 L858R mutation
Maemondo et al. [18]	2010	NA	IIIB/IV	228	Gefitinib	CTX	Exon 19 deletion or exon 21 L858R mutation
Mitsudomi et al. [19]	2010	III	IIIB/IV	177	Gefitinib	CTX	Exon 19 deletion or exon 21 L858R mutation
Han et al. [20]	2017	II	IIIB/IV	121	Gefitinib	CTX	Exon 19 deletion or exon 21 L858R mutation
Patil et al. [21]	2017	III	IIIB/IV	290	Gefitinib	CTX	Exon 19 deletion or exon 21 L858R mutation
Sequist et al. [22]	2013	III	IIIB/IV	345	Afatinib	CTX	Exon 19 deletion or exon 21 L858R mutation or others
Wu et al. [23]	2014	III	IIIB/IV	364	Afatinib	CTX	Leu858Arg, exon 19 deletions, or other
Lynch et al. [24]	2010	III	IIIB/IV	676	Cetuximab	CTX	N/A
Pirker et al. [25]	2009	III	IIIB/IV	748	Cetuximab	CTX	N/A
Shi et al. [26]	2017	III	IIIB/IV	285	Icotinib	CTX	Exon 19/21 EGFR mutations

## Data Availability

All data generated or analyzed during this study are included in this published article.
